# Biaxial Estimation of Biomechanical Constitutive Parameters of Passive Porcine Sclera Soft Tissue

**DOI:** 10.1155/2022/4775595

**Published:** 2022-02-28

**Authors:** Zwelihle Ndlovu, Dawood Desai, Thanyani Pandelani, Harry Ngwangwa, Fulufhelo Nemavhola

**Affiliations:** ^1^Unisa Biomedical Engineering Research Group, Department of Mechanical Engineering, School of Engineering, College of Science Engineering and Technology, University of South Africa, Pretoria 0001, South Africa; ^2^Department of Mechanical and Mechatronics Engineering, Faculty of Engineering and Built Environment, Tshwane University of Technology, South Africa; ^3^Council for Scientific and Industrial and Research, Defence and Security Cluster, Brummeria, Pretoria 0001, South Africa

## Abstract

This study assesses the modelling capabilities of four constitutive hyperelastic material models to fit the experimental data of the porcine sclera soft tissue. It further estimates the material parameters and discusses their applicability to a finite element model by examining the statistical dispersion measured through the standard deviation. Fifteen sclera tissues were harvested from porcine' slaughtered at an abattoir and were subjected to equi-biaxial testing. The results show that all the four material models yielded very good correlations at correlations above 96%. The polynomial (anisotropic) model gave the best correlation of 98%. However, the estimated material parameters varied widely from one test to another such that there would be need to normalise the test data to avoid long optimisation processes after applying the average material parameters to finite element models. However, for application of the estimated material parameters to finite element models, there would be need to consider normalising the test data to reduce the search region for the optimisation algorithms. Although the polynomial (anisotropic) model yielded the best correlation, it was found that the Choi-Vito had the least variation in the estimated material parameters, thereby making it an easier option for application of its material parameters to a finite element model and requiring minimum effort in the optimisation procedure. For the porcine sclera tissue, it was found that the anisotropy was more influenced by the fiber-related properties than the background material matrix-related properties.

## 1. Introduction

It is reported that majority of the vision impairment may be prevented or treated if caught early, and correct therapies are implemented. Globally, 86.1 million cases leading to the moderate and severe vision impairment were caused by undercorrected refractive error. Due to increase in aging population in many countries across the globe, vision impairment including uncorrected refractive error, glaucoma, and contract were reported to be in the rise. The rise in vision impairment is due to rising sociodemographic status and life expectancy witnessed in number of countries globally [1–4]. It is reported that 4.8 million and 21.4 million people are blind and visually impaired in 48 countries of sub-Saharan Africa [5]. In addition, Africa has been reported to be carrying approximately 19% of the global blindness [6]. Blindness prevalence rates vary widely but the evidence suggests that approximately 1% of people in sub-Saharan Africa are blind [7]. Visual impairment is a significant health problem in the sub-Saharan Africa. The major eye conditions include cataracts, uncorrected refractive errors, glaucoma, age-related macular degeneration, corneal opacities, diabetic retinopathy, trachoma, and onchocerciasis [8, 9]. In addition, glaucoma is labelled as worldwide problem of the eye diseases where 111 million of individuals are projected to be affected by 2040 [10]. Therefore, it is vital that the biomechanical properties and computational models of the eye soft tissues are developed with the view to understand the mechanisms of various diseases of the eye. Biomechanical properties of eye soft tissues are vital in improving insight into how eye diseases progress [11].

Biomechanical properties of the soft tissues have been utilised previously to study mechanical behaviour [12–14]. The progression of the diseases was also studied by developing accurate and reliable computational models [15, 16]. The detailed computational models of the eye request a thorough study of mechanical properties including the fitting of constitutive hyperelastic models. Previously, different biomechanical properties of the different ocular tissues including sclera [17–19], orbital connective tissue and fat [20, 21], cornea [22–24], and extraocular muscles [25, 26]. Sclera is normally associated with near-sightedness (myopia), and therefore, there is considerable amount of work done on the investigation of the biomechanical properties of sclera [27, 28]. In particular, the mechanical properties of the sclera are critical for the development of synthetic materials for the replacement of eye tissues. This is because globally, there is a rise of accident where organ such as eye may be lost or damaged permanently. In our previous studies, we presented the biaxial mechanical characterisation of the sheep sclera soft tissue [28]. In this study, the Fung and Choi-Vito hyperelastic constitutive models were fitted on the biaxial tensile data. Finite element modelling (FEM) has been previously utilised in studying how soft tissues behave under mechanical loading [29–35]. These constitutive parameters generated by fitting biaxial tensile data may be utilised for detailed study of diseases' progression in the eye as well as understanding pain dissemination based on the needle injection in the sclera for treatment [36, 37].

In this study, we present the biaxial biomechanical properties of the porcine sclera soft tissue. The porcine anatomy has been reported to be like that of human beings; therefore, it is believed that the biaxial mechanical data presented in this study will be useful for studying human eye diseases. Therefore, the aim of this study is to generate constitutive parameters of the porcine sclera soft tissues subjected to equi-biaxial loading. Fung, Choi-Vito, Holzapfel (2000), and polynomial (anisotropic) hyperelastic constitutive models are fitted in the equi-biaxial tensile data to estimate the constitutive material parameters. To our knowledge, there is no study that looked at utilising and comparing the Fung, Choi-Vito, Holzapfel (2000), and polynomial (anisotropic) hyperelastic constitutive models in estimating the material parameters of the porcine sclera soft tissue.

## 2. Methods and Materials

### 2.1. Sample Preparation

The sample consists of sclera (*N* = 15) soft tissue harvested from the local abattoir with unknown ages and sexes. To preserve the mechanical properties of the sclera soft tissue, the specimen was collected within 4 to 6 hours after slaughter as discussed [38]. The detailed tissue preparation of the porcine sclera is like what we have previously presented [28]. To avoid possible deterioration of the sclera tissue including dehydration, specimen was placed in ice bag on the way to the Unisa Biomechanics Laboratory. During further processing, the unwanted ocular tissues were removed from the porcine eye using surgical blades. Two square samples of 12 × 12 mm (Figure 1) were cut from each eye roughly 4 to 6 mm away from the optic nerve head and corneal limbus to reduce thickness variation. Vernier caliper was then utilized to measure the thickness of the sclera tissue. Randomly, the thickness of the sclera tissue was measured in four different places, and the average thickness was taken for further processing of the data. Specimens were subjected to visual inspection before individually subjected to biaxial testing equipment. Reason for visual inspection was to ensure that there was no physical damage on the tissue that may influence the mechanical data. Samples were dipped and kept in isotonic solution 9.0 g/l at pH of 5.5 for about 15 to 20 minutes before testing.

### 2.2. Mechanical Testing

Biaxial mechanical properties of the porcine sclera soft tissue were captured using custom-built biaxial testing device, Bio-Tester 5000 from Cellscale (Waterloo, Canada) with load capacity of 23000 mN and accuracy of 5000 *μ*N (Figure 2). CellScale BioRakes were utilized to clamp the sclera soft tissue on all sides when equi-biaxial strain is applied. Strain rate of between 0.452 mm/s was applied during biaxial testing of each sample. To mimic the body temperature, the water bath was heated to 37°C. The temperature sensor is integrated in the custom-built biaxial device to ensure that the temperate is kept constant through testing. *X* and *Y* directions were considered as circumferential and longitudinal directions, respectively. Four (4) CellScale BioRakes were used to mount the specimens to develop mechanical properties. On both *x* and *y* directions, all fifteen (15) specimens were subjected to 25% strain using only strain-controlled mode equally in both directions.

## 3. Theoretical Framework

### 3.1. Tissue Stress-Strain Analysis

In this study, the stresses were calculated through the first Piola-Kirchoff stress *T* in the two directions using the equation:

(1) $$\begin{array}{c} T_{ii}=\frac{F_{ii}}{L_{i0}h_{0}}, \end{array}$$

where *F* is the load vector in directions *i* = 1, 2, and for the current study, these indices represent longitudinal (cross-fiber-direction) and circumferential (fiber-direction) direction. The index 0 denotes the undeformed state. *L* represents tissue length, and *h* represents tissue thickness.

The finite strains were calculated by the formula:

(2) $$\begin{array}{c} \varepsilon_{i}=\frac{L_{i}-L_{i0}}{L_{i0}}. \end{array}$$

The stress results in Equation (1) are however noisy; therefore, they were further filtered with an 8-point moving average filter in Excel. The data were resampled and further smoothened using a quadratic function.

### 3.2. Constitutive Modelling

The passive response of a biological soft tissue is more complex than the response of elastic solids due to the fact that they undergo finite deformations under mechanical loads [39, 40]. Thus, the passive phases of tissues' deformations are considered using the nonlinear theory of hyperelasticity. The most useful quantity in deriving the expressions for the passive response of materials that undergo finite deformation is the strain energy function [40]. There is a huge number of variations of its implementation in the literature depending on different cases. In this study, we assume that the tracheal tissue is anisotropic and incompressible; therefore, we apply and study the material parameters from six models, namely, the Fung, Choi-Vito, Holzapfel (2000), and polynomial (anisotropic) models. In the following sections, these models are presented in terms of their strain energy functions.

#### 3.2.1. The Fung Model

The Fung model is a hyperelastic anisotropic material model for stress-strain description of arterial wall. It is phenomenological in nature and its incompressible form is given by [41].

(3) $$\begin{array}{c} W=\frac{c}{2}\left(e^{Q}-1\right),\\ Q=b_{1}E_{\theta \theta }^{2}+b_{2}E_{ZZ}^{2}+b_{3}E_{RR}^{2}+2b_{4}E_{\theta \theta }E_{ZZ}+2b_{5}E_{ZZ}E_{RR}+2b_{6}E_{RR}E_{\theta \theta }, \end{array}$$

where *E*_*ij*_(*i*, *j* = *θ*, *Z*, *R*) are the Green strain components and (*θ*, *Z*, *R*) are the cylindrical coordinates in the radial, circumferential, and axial reference directions, respectively. *c* stress-like material parameter and *b*_*i*_ are the nondimensional material parameters.

#### 3.2.2. Choi-Vito Model

Choi-Vito model is hyperelastic anisotropic material model developed for canine pericardium. The model is fully phenomenological and formulated through the components of Green-Lagrange strain tensor. The model is implemented in an exponential format, and its strain-energy function is expressed as [42]

(4) $$\begin{array}{c} W=b_{0}\left[\exp\left(b_{1}E_{\theta \theta }^{2}\right)+\exp\left(b_{2}E_{ZZ}^{2}\right)+\exp\left(2b_{3}E_{\theta \theta }E_{ZZ}\right)-3\right], \end{array}$$

where *b*_*i*_ are the material parameters.

#### 3.2.3. The Holzapfel (2000) Model

This model is hyperelastic anisotropic material model for stress-strain description of arterial layers. It is constituted by forms of the strain energy function that represent isotropy and anisotropy. Thus, its strain energy function is given by [43].

For incompressible formulation:

(5) $$\begin{array}{c} W_{f\left(I_{1,}I_{4},I_{6}\right)}=\frac{\mu }{2}\left(I_{1}-3\right)+\frac{c_{1}}{2c_{2}}\underset{i=4,6}{\sum }\left(\exp^{c_{2}{\left(I_{i}-1\right)}^{2}}-1\right), \end{array}$$

where the constant *μ* is associated with the noncollagenous matrix of the material, which describes the isotropic part of the overall response of the tissue. The constants *c*_1_ and *c*_2_ are associated with the anisotropic contribution of collagen to the overall response of the tissue. The material parameters are constants and do not depend on the geometry, opening angle, or fiber angle. The model is implemented in an exponential format, and *I*_1_, *I*_4_, and *I*_6_ are (pseudo-) invariants of **C** (**G**_0_ and **H**_0_). **G**_0_, **H**_0_ are structural tensors referenced to individual family of fibers.

#### 3.2.4. The Polynomial (Anisotropic) Model

Like its name, this model is hyperelastic anisotropic material model whose strain energy function is expressed as a polynomial series of isotropic and anisotropic strain invariants given as [44]

(6) $$\begin{array}{c} W=\overset{3}{\underset{i=1}{\sum }}a_{i}{\left(I_{1}-3\right)}^{i}+\overset{3}{\underset{j=1}{\sum }}b_{j}{\left(I_{2}-3\right)}^{j}+\overset{6}{\underset{k=2}{\sum }}c_{k}{\left(I_{4}-1\right)}^{k}+\overset{6}{\underset{m=2}{\sum }}e_{m}{\left(I_{6}-1\right)}^{m}, \end{array}$$

where *a*_*i*_, *b*_*j*_, are stress-like material parameters referenced to isotropic (matrix) properties. *c*_*k*_, and *e*_*m*_ are stress-like material parameters referenced to anisotropic (fiber) properties. *I*_1_, *I*_2_, *I*_4_, and *I*_6_ are (pseudo-)invariants of *C* (**A**_0_ and **B**_0_). **A**_0_, **B**_0_ are structural tensors referenced to individual family of fibers. **C** is right Cauchy-Green definition tensor.

The four material models are classified further according to the type of material parameters that they represent in Table 1. From the table, the models can be grouped into two main classes: those that model the soft tissue as layers of general material matrix and those that model the soft tissue as composite material with embedment of fiber structures within the layers of material matrix. These models may also be classified into purely phenomenological or structural scenario. Material parameter defining the orientation angle of fibers (measured from axis “1”) in the undeformed configuration is included in the analysis. In this analysis, both the *x* and *y* directions were plotted simultaneously including the fibre angle term.

### 3.3. Data Analysis

In this study, we use the constrained optimisation by linear approximation algorithm (COBYLA (3^rd^ party: SciPy)) implemented in Hyperfit software for fitting the equi-biaxial tensile experimental data of Fung, Choi-Vito, Holzapfel (2000), and polynomial (anisotropic) hyperelastic constitutive models given in Equations (3)–(6). The coefficient of determination, *R*^2^, which measures the correlation of one variable with another, is evaluated for each model. The coefficient of determination (*R*^2^) (also known as Nash-Sutcliffe coefficient) is defined as follows [45–47]:

(7) $$\begin{array}{c} R^{2}=1-\frac{\sum_{i=1}^{n}{\left(y_{e}-y_{m}\right)}^{2}}{\sum_{i=1}^{n}{\left(y_{e}-\bar{y_{e}}\right)}^{2}}, \end{array}$$

where *y*_*e*_ is the experimental data, *y*_*m*_ is the model predicted data, $\bar{y_{e}}$ is the average value of the experimental data, the indices *i*, ⋯, *n* denote the data points, and *R*^2^*ϵ*〈−∞, 1〉, where a perfect fit is defined for *R*^2^ = 1.

## 4. Results

Stress-strain curves for the porcine sclera soft tissue subjected to equi-biaxial tensile loading are plotted in Figure 3. The stress-strain curves for porcine sclera soft tissue show that the tissue has a well-defined nonlinear behaviour as the tissue gets stretched from the toe region to 25% strain.

This study is aimed at estimating the biomechanical material parameters of a porcine sclera using four different constitutive material models, namely, Fung, Choi-Vito, Holzapfel (2000), and polynomial (anisotropic) models. All the above material models are hyperelastic anisotropic models which employ different modelling frameworks as presented in Equations (3)–(6) in Section 3.2. The material parameters for each model for all the fifteen tests are given in Tables 2–4. The tabulated results show that all the models yield very good correlations at greater than 96% with standard deviations of less than 3.2%. This implies that the model predictions were very close to the mean stress-strain curves for all the four models in this study.

However, the polynomial (anisotropic) model yielded the best correlation at an average of 98.3% and an average standard deviation of approximately 1.73%, while the Fung model yielded the lowest average correlation of 96.4% with an average standard deviation of 3.2%. The Choi-Vito and Holzapfel models had similar average correlations of 97.2% with average standard deviations of 1.65% and 2.98%, respectively.

In terms of statistical dispersion in the estimated material parameters by the four models, the polynomial (anisotropic) model had the largest variance with the widest scatter in the material parameters over the fifteen different tests. An evaluation of the standard deviation percentage yielded deviations from 110% to 660% for the polynomial (anisotropic) model. On the other hand, the Choi-Vito model had the smallest variance in the material parameters with deviations between 31% and 91%. This result might not be surprising considering that the Choi-Vito model was originally formulated for the pericardium tissue [42, 48, 49] which, in much respect, may be similar in functionality to the sclera tissue. The implications of such deviations in terms of applying the estimated average material parameters directly to finite element (FE) models is problematic, and this has been discussed in the next section. From Figure 4, the polynomial (anisotropic) constitutive model yields the highest *R*^2^ of 0.983 while the Fung constitutive model yields the lowest *R*^2^ of 0.964. On the other hand, Figure 5 shows that the porcine sclera soft tissue was found to be much stiffer in the circumferential direction with stress values taken at 15% strain.

## 5. Discussion

The results of correlations between model predictions and tests presented in Section 4 should never be taken at face value. It should be noted that a model is applied to a given set of experimental data from which the material parameters are estimated. Thus, each material model is optimised for each fresh set of experimental data with totally different target values, and therefore, it is likely to yield material parameters that are different from those obtained from the other tests. This is where some form of calibration may become necessary to eliminate huge variances in the model parameters from one test to another [50–53]. Dubuis et al. [54] employed a calibration technique in which the FE itself was calibrated using 3D CT scans.

Therefore, in applying the average material parameters obtained here to an FE model, one may need to consider implementing an optimisation procedure in which these average values may be used as seed values [55]. Kollmann et al. [55] applied such methods for optimisation of the parameters used in FE modelling of asphalt mixtures. For models with large numbers of material parameters such as the polynomial (anisotropic) model in this study, it might be prudent to conduct an initial sensitivity analysis to determine the most influential material parameters. Biaxial tensile testing has been utilised in understanding the mechanical properties of soft tissues. Additionally, hyperelastic constitutive models have also been presented by fitting the constitutive models of the various soft tissues including heart myocardium [56–58] and omasum [59].

Despite the highest correlation obtained for the polynomial (anisotropic) model, the direct application of its parameters to an FE model can yield huge errors due to the wide scatter of its material parameters. One may need to prescribe huge range of its parameter space within which the optimisation algorithm can search for the optimal material parameters to give accurate correlation for any given random test. Among the four material models in this study, the Choi-Vito model offers the best chance for attaining accurate correlations when directly applied to an FE model with minimal effort of optimisation. For the Choi-Vito model, only the stress-like material parameter may take more time in searching for optimal material parameter at 91% deviation from the mean value. Apart from the average value given in Table 3, the other best value from which to start the search for the stress-like material parameter for the Choi-Vito may be the gradient of the linear elastic portion of the stress-strain curve.

In terms of general material matrix anisotropy, both the Fung and Choi-Vito models do not show that the porcine sclera tissue is heavily anisotropic between the circumferential and longitudinal direction. However, the tissue seems to be different in material matrix in the radial direction from the Fung model. The values of *a*_*i*_ and *b*_*j*_ which also represent the material matrix properties in the polynomial (anisotropic) model show that there is no significant anisotropy between the circumferential and longitudinal directions. On the other hand, the *c*_*k*_ material parameters in the polynomial (anisotropic) model and the *k*_*i*_ parameters in the Holzapfel (2000) model, all of which represent material parameters related with fiber properties, exhibit significant anisotropy in Tables 5 and 4. This implies that the anisotropy in the porcine sclera tissue is mainly due to different fiber properties between the circumferential and longitudinal directions and not the background material matrix properties. It is difficult to establish in this study if the fiber orientation angle had any influence on the accuracy of the correlations in the polynomial (anisotropic) and Holzapfel (2000) models. This can be better investigated through the sensitivity analysis.  Table 6 shows the box plot properties of the coefficient of determination (*R*^2^) having *Q*1, median, and *Q*3. It is clear from the table that the four models have approximately equal coefficients of determination with the Fung and Holzapfel (2000) models exhibiting the largest and lowest ranges in the *R*^2^ values as represented by the IQR values.

## 6. Conclusion

The study applies four different hyperelastic material models to estimate the material parameters for the computational modelling of porcine sclera tissue. It is found that all the four material models produce very good correlations higher than 96% with the polynomial (anisotropic) model yielding the highest correlation of 98%. However, the variation of the material parameters from one test to another is a challenge as far as their direction application to FE models is concerned. For example, the polynomial (anisotropic) model has the minimum standard deviation of its material parameters from one test to another as 110%. Thus, the average material parameters obtained in this paper may result in inaccurate correlations in the FE predicted results. One way to deal with this challenge is to implement an optimisation routine which uses these material parameters as seed values. However, with such large spread in the parameter space, the search algorithm may take too long to converge especially with material models that have large numbers of estimated material parameters. Therefore, it is proposed that the test data should also be normalised or calibrated before application of the constitutive material models to reduce the variation in the estimated parameters thereby reducing the search region. In this study it is also found that the Choi-Vito model has the least variation in its material parameters. Thus, it might offer much better chance than the other models for convergence to material parameters that can yield very good correlations for the FE model. In terms of the models that are based on fiber-property formulation as identified in Table 1, the Holzapfel (2000) model offers a better option as compared to the polynomial (anisotropic) model for faster convergence as its material variation is much lower between the two models. As far as anisotropy in the porcine sclera tissue is concerned, both the polynomial (anisotropic) model and the Holzapfel (2000) model show that the fiber properties have more influence than the background material matrix. It is not clear if the angle of fiber orientation has any influence in the results. This might require more investigation.

## 7. Limitation

The limitation of this experimental study is that it did not segment porcine sclera per region. The thickness of porcine sclera samples used in this work was unknown. This may lead to unclear results since it was reported that some regions in the sclera exhibit anisotropy while others do not. However, it has been reported that porcine and human sclera behave in the same way despite a difference in tissue thickness. The two tissues are similar in terms of structure, histology, and collagen fiber architecture and should have similar material properties and will be useful for studying human eye diseases [60].

No imaging/microscopy was done in this study; hence, the fiber direction cannot be determined with certainty. It has previously been observed that the porcine sclera has a blood vessel that travels parallel to the ora serrata [61]. This vessel could introduce stiffening of one fiber direction and can result in different material properties compared to another fiber direction.

Further studies should be conducted to confirm human and porcine similarities with regard to material properties. Porcine sclera is easily available and can be an efficient substitute for human sclera material properties, in computational modelling.

## Figures and Tables

**Figure 1:** Porcine sclera tissue samples (a) cut from each eye immediately after the delivery from the abattoir to the Unisa Biomechanics Laboratories with a sketch showing how the tissue was excised from the porcine eye (b). The reference axis were defined in such a way that the longitudinal direction is from the cornea to the base while circumferential direction is 90° with the longitudinal direction.

**Figure 2:** Experimental set-up of porcine sclera tissue subjected to biaxial tensile loading (Bio-Tester 5000 from Cellscale) (Waterloo, Canada). The hooks (BioRakes) were utilised in securing the sclera tissue and were punched thoroughly before they were inserted into the warm bath of isotonic solution 9.0 g/l at pH of 5.5 at a temperature of 37°C.

**Figure 3:** Porcine sclera soft tissue (*N* = 18) subjected to equi-biaxial mechanical forces showing stress (kPa) vs. strain mechanical properties up to 25% strain (a) circumferential and (b) longitudinal. Test 3 and test 4 are showing the lowest and highest tress in the circumferential direction, respectively. Additionally, test 1 is showing the highest stress, and test 15 is showing the lowest stress in the longitudinal direction, respectively.

**Figure 4:** Average coefficient of determination (*R*^2^) (with standard error) of the porcine soft tissue sclera calculated for Holzapfel (2000), Choi-Vito, Fung, and polynomial (anisotropic) hyperelastic constitutive models, with polynomial (anisotropic) constitutive model showing the highest *R*^2^ of 0.983 and the lowest *R*^2^ of 0.964 observed for Fung constitutive model.

**Figure 5:** First Piola-Kirchhhoff stress (kPa) values taken at 15% engineering strain of the porcine soft tissue subjected to biaxial tension in two loading directions: (a) longitudinal and (b) circumferential.

**Table 1:** The classification of the four hyperelastic anisotropic material models according to the material properties they represent. The Fung and Choi-Vito are classified as the models that model the soft tissue as layers of general material matrix, while the polynomial (anisotropic) and Holzapfel (2000) models are those that model the soft tissue as composite material with embedment of fiber structures within the layers of material matrix.

Model	Stress-like material parameter	Dimensionless material parameter	Stress-like material parameter referred to material matrix property	Stress-like material property referred to fiber property	Dimensionless material property referred to fiber property	Material parameter referred to fiber angle orientation
Polynomial (anisotropic)			✓ (*a*_*i*_, *b*_*j*_)	✓ (*c*_*k*_)		✓ (*φ*)
Fung	✓ (*c*)	✓ (*b*_*i*_, *i* = 1 ⋯ 6)				
Choi-Vito	✓ (*b*_0_)	✓ (*b*_*i*_, *i* = 1 ⋯ 3)				
Holzapfel 2000			✓ (*μ*)	✓ (*c*_1_)	✓ (*c*_2_)	✓ (*φ*)

**Table 2:** Estimated material parameters of porcine sclera soft tissue loaded biaxially using Fung hyperelastic constitutive model including the coefficient of determination (*R*^2^) of each specimen (*N* = 15). The average constitutive (*c*, *b*_1_, *b*_2_, *b*_3_, *b*_4_, *b*_5_, *b*_6_, and *R*^2^) parameters are also included.

Test #	*R* ^2^	*c*	*b*_1_	*b*_2_	*b*_3_	*b*_4_	*b*_5_	*b*_6_
S1	0.985	1.527	1.264	1.228	-0.655	0.375	0.243	0.329
S2	0.959	1.533	0.952	1.139	-0.420	0.460	0.569	-0.027
S3	0.993	1.050	1.200	1.178	-0.118	0.533	0.379	0.628
S4	0.900	0.137	3.965	1.971	-1.625	2.864	1.851	-1.999
S5	0.971	0.500	1.924	2.824	-0.643	1.242	1.147	0.739
S6	0.907	0.791	1.293	0.801	-0.345	1.038	0.630	0.289
S7	0.915	0.822	3.911	1.877	1.002	2.527	2.473	0.068
S8	0.957	0.929	1.299	0.902	-0.388	1.071	0.563	0.513
S9	0.993	0.558	2.701	3.301	1.488	3.039	2.612	2.439
S10	0.983	0.158	4.686	3.439	-0.125	2.827	1.727	2.578
S11	0.960	0.960	1.102	0.808	-0.130	0.298	0.297	0.260
S12	0.983	1.286	1.000	0.857	-0.335	0.390	0.265	0.283
S13	0.990	1.286	1.671	0.601	-0.280	1.123	0.507	0.614
S14	0.983	1.026	0.976	1.200	-0.374	1.074	0.635	0.465
S15	0.984	0.910	1.517	0.679	-0.318	1.111	0.442	0.546
Average	**0.964**	**0.898**	**1.964**	**1.520**	**-0.218**	**1.331**	**0.956**	**0.515**
STD	**0.031**	**0.413**	**1.202**	**0.921**	**0.679**	**0.949**	**0.783**	**1.002**

**Table 3:** Estimated material parameters of porcine sclera soft tissue loaded biaxially using Choi-Vito hyperelastic constitutive model including the coefficient of determination (*R*^2^) of each specimen (*N* = 15). The average constitutive (*c*, *b*_1_, *b*_2_, *b*_3_, and *R*^2^) parameters are also included.

Test #	*R* ^2^	*c*	*b*_1_	*b*_2_	*b*_3_
S1	0.979	0.004	3.180	11.421	39.018
S2	0.956	0.006	-2.627	10.015	21.673
S3	0.967	0.011	21.724	26.703	11.276
S4	0.985	0.017	39.952	17.770	9.632
S5	0.981	0.024	23.364	27.074	17.790
S6	0.935	0.011	47.858	17.579	6.936
S7	0.974	0.012	40.348	14.985	14.470
S8	0.976	0.018	36.901	25.357	14.662
S9	0.990	0.022	29.680	34.177	23.643
S10	0.983	0.029	17.587	16.756	15.163
S11	0.981	0.015	27.327	19.054	2.194
S12	0.985	0.039	20.816	18.381	13.656
S13	0.969	0.036	34.998	18.118	15.893
S14	0.994	0.093	14.175	14.101	13.318
S15	0.946	0.024	31.969	14.387	2.134
Average	**0.972**	**0.023**	**26.141**	**20.467**	**15.324**
STD	**0.016**	**0.021**	**13.494**	**6.348**	**8.741**

**Table 4:** Estimated material parameters of porcine sclera soft tissue loaded biaxially using Holzapfel (2000) hyperelastic constitutive model including the coefficient of determination (*R*^2^) of each specimen (*N* = 15). The average constitutive (*c*, *b*_1_, *b*_2_, *b*_3_, and *R*^2^) parameters are also included.

Test #	*R* ^2^	*μ*	*k*_1_	*k*_2_	*φ*
S1	0.982	0.000	0.039	9.303	0.814
S2	0.972	0.000	0.036	5.250	2.240
S3	0.984	0.000	0.098	6.017	-0.389
S4	0.974	0.000	0.059	7.572	0.856
S5	0.864	0.068	0.048	7.676	0.311
S6	0.976	0.000	0.052	6.142	-0.362
S7	0.980	0.000	0.081	6.658	0.630
S8	0.983	0.000	0.077	8.141	0.854
S9	0.975	0.000	0.042	5.971	0.755
S10	0.978	0.000	0.078	3.696	0.649
S11	0.978	0.000	0.091	4.981	0.723
S12	0.980	0.000	0.116	7.329	0.457
S13	0.980	0.000	0.078	7.284	0.778
S14	0.982	0.013	0.083	8.418	0.549
S15	0.990	0.000	0.101	3.848	0.854
Average	**0.972**	**0.005**	**0.074**	**6.767**	**0.654**
STD	**0.029**	**0.017**	**0.024**	**2.263**	**0.562**

**Table 5:** Estimated material parameters of porcine sclera soft tissue loaded biaxially using polynomial (anisotropic) hyperelastic constitutive model including the coefficient of determination (*R*^2^) of each specimen (*N* = 15). The average constitutive (*a*_1_, *a*_2_, *a*_3_, *b*_1_, *b*_2_, *b*_3_, *c*_2_, *c*_3_, *c*_4_, *c*_5_, *c*_6_, *φ*, and *R*^2^) parameters are also included.

	*R* ^2^	*a*_1_	*a*_2_	*a*_3_	*b*_1_	*b*_2_	*b*_3_	*c*_2_	*c*_3_	*c*_4_	*c*_5_	*c*_6_	*φ*
S1	0.953	0.045	0.014	0.035	-0.002	-0.003	-0.002	-0.027	-0.007	-0.018	-0.010	0.994	0.944
S2	0.976	0.023	0.048	0.039	0.000	0.001	-0.005	-0.015	0.001	0.006	0.010	0.022	0.003
S3	0.983	-0.011	0.102	-0.072	-0.220	-0.089	-0.133	-0.005	0.074	0.201	0.174	-0.259	0.268
S4	0.954	0.018	0.055	-0.051	0.035	0.031	0.021	0.011	-0.022	-0.041	-0.040	1.217	0.911
S5	0.948	0.006	0.216	-0.302	-0.095	-0.042	0.007	-0.039	0.150	0.035	0.050	-0.011	0.016
S6	0.990	0.010	-0.016	0.074	0.233	-0.158	0.186	-0.008	-0.018	0.247	0.394	-0.825	-0.083
S7	0.997	0.014	0.007	0.298	-0.118	-0.285	-0.112	-0.038	0.245	-0.217	-0.004	-0.019	0.199
S8	0.998	0.003	0.225	0.206	-0.305	0.319	-0.283	0.006	-0.096	0.195	-0.325	0.310	-0.089
S9	0.991	0.004	0.087	0.039	0.012	-0.082	0.026	-0.005	-0.006	0.024	0.016	0.015	-0.056
S10	0.993	0.015	0.093	0.006	-0.043	0.008	-0.004	0.000	-0.046	0.154	0.048	-0.147	-0.085
S11	0.998	0.008	0.201	-0.061	-0.425	0.155	0.060	-0.012	0.020	0.081	-0.155	0.180	0.216
S12	0.989	0.028	-0.011	0.075	-0.289	-0.477	-0.220	-0.004	0.003	0.465	0.198	-0.928	0.460
S13	0.989	0.028	-0.011	0.075	-0.289	-0.477	-0.220	-0.004	0.003	0.465	0.198	-0.928	0.460
S14	0.992	-0.013	0.081	-0.707	0.254	-0.952	0.325	0.031	-0.058	0.762	0.610	-4.150	0.592
S15	0.991	-0.001	0.375	-0.293	0.335	-0.371	0.014	-0.003	-0.032	-0.166	0.269	0.152	0.081
Average	**0.983**	**0.012**	**0.098**	**-0.043**	**-0.061**	**-0.161**	**-0.023**	**-0.007**	**0.014**	**0.146**	**0.096**	**-0.292**	**0.256**
STD	**0.017**	**0.015**	**0.108**	**0.233**	**0.215**	**0.301**	**0.152**	**0.017**	**0.082**	**0.250**	**0.217**	**1.185**	**0.337**

**Table 6:** Fitting of hyperelastic models (*N* = 15) showing box plot properties of the coefficient of determination (*R*^2^) with *Q*1, median, and *Q*3 values.

	Polynomial model	Fung model	Choi-Vito model	Holzapfel (2000) model
Min	0.948	0.900	0.935	0.864
*Q*1	0.980	0.958	0.968	0.976
Median	0.990	0.983	0.979	0.980
*Q*3	0.993	0.985	0.984	0.982
Max	0.998	0.993	0.994	0.990
IQR	0.013	0.027	0.016	0.006

## Data Availability

All data is available in the main manuscript.

## Additional Points

Correspondence and requests for materials should be addressed to F.N. Reprints and permissions information is available at http://www.nature.com/reprints.
